The article "Correlation between Platelet miRNA Expression and Coagulation Function in Children with Severe Pneumonia" was retracted in 2023. Reasons: signs of a paper mill; compromised peer review; unreliable results or conclusions.

# Correlation between Platelet miRNA Expression and Coagulation Function in Children with Severe Pneumonia

**DOI:** 10.1155/2022/2826115

**Published:** 2022-06-22

**Authors:** Mingming Hao, Jing Guo, Jinying Lu, Taotao Chang, Zhanru Yin

**Affiliations:** Department of Pediatrics, Hengshui People's Hospital, Hengshui, Hebei, China

## Abstract

**Objective:**

To investigate the relationship between expression levels of platelet miRNAs and severe pneumonia (SP) in children.

**Methods:**

A randomized controlled trial was conducted in 129 children with SP hospitalized from May 2018 to May 2020. All children joined the study group and were divided into the mild infection group, moderate infection group, and severe infection group according to the diagnostic criteria, 43 cases in each group. Besides, 129 healthy children were selected as the control group. The expression levels of platelet miR-223 and miR-192 were detected by real-time quantitative polymerase chain reaction (qPCR). The prothrombin time (PT), activated partial thromboplastin time (APTT), and fibrinogen (FIB) were detected by the Sysmex CA-1500 System (Sysmex Corporation, Japan). The Pearson analysis was conducted to evaluate the correlation between coagulation function and the levels of miR-223 and miR-192.

**Results:**

Compared with the control group, miR-223 in the study group was significantly higher and miR-192 was significantly lower (*P* < 0.05). Compared with the mild infection group, miR-223 was significantly higher and miR-192 was significantly lower in the moderate infection group and severe infection group (*P* < 0.05). Compared with the control group, PT and APTT were significantly lower and FIB was significantly higher in the study group (*P* < 0.05). Pearson correlation analysis revealed that miR-223 was positively correlated with PT and APTT (*P* < 0.05) and negatively correlated with FIB (*P* < 0.05); miR-192 was negatively correlated with PT and APTT (*P* < 0.05) and positively correlated with FIB (*P* < 0.05).

**Conclusion:**

miR-223 and miR-192 can reflect coagulation function in children with SP, which can provide a certain reference basis for clinical guidance and treatment and prognosis.

## 1. Introduction

Pneumonia, as one of the respiratory tract infection diseases, is endemic in children, especially infants [1]. Pneumonia is divided into mild type and severe type based on its severity. Mild type has a good prognosis and few complications with low mortality. Due to the rapid onset, severity, and rapid development, severe type has more complications, even life-threatening. It is be identified as the main cause of death in children under 5 years of age [2]. Severe pneumonia (SP) accounts for about 8–14% in children with pneumonia, and failure to control timely and effectively can lead to multiple organ dysfunction syndrome (MODS) and septic shock [3]. The disease is complex and changeable and even complicated by respiratory failure, which seriously affects the physical and mental health. Therefore, it is particularly important to take active and correct treatment methods in clinical practice. In recent years, research reports have shown that children with severe pneumonia have achieved significant clinical effects with integrated traditional Chinese and Western medicine. Therefore, early diagnosis and effective treatment of SP in children is an important component in pediatrics. miRNA, a class of highly conserved endogenous noncoding single-stranded RNA with a length of 21–25 nt, regulates factors at the gene expression level after transcription and mediates gene silencing after transcription [4]. miRNA participates in many biological processes such as metabolism, cell differentiation, apoptosis, and disease control. They are involved in multiple systems including respiratory, cardiovascular, nervous, and hematopoietic systems. A previous study has reported that miRNA is involved in angiogenesis and erythropoiesis [5]. Data from several studies suggest that miRNA is strongly associated with the occurrence, development, and outcome of pulmonary diseases and has gradually become a reliable biomarker in the diagnosis of diseases [6, 7]. But the publications that concentrate on the relationship of miRNA and coagulation function in children with SP are few.

Here, we conducted the study to investigate the relationship of miRNA and coagulation function in children with SP.

## 2. Materials and Methods

### 2.1. General Materials

A total of 129 children with pneumonia up in hospital from May 2018 to May 2020 were selected as the study group, 69 males and 60 females with an age of (3.62 ± 1.21) years. The children were divided into the mild infection group, moderate infection group, and severe infection group, according to the diagnostic criteria, 43 cases in each group. Besides, 129 healthy children up in hospital for physical examination during the same period were selected as the control group, 70 males and 59 females with an age of (3.66 ± 1.24) years. They were free of chronic disease and had experienced no acute infectious disease within 6 weeks. Further statistical tests revealed no significant differences in general materials (*P* > 0.05). The informed consent process follows regulations; the legal representative of the children signed the informed consent files. The studies involving human participants were reviewed and approved by Hengshui People's Hospital, no. HSP77738.

### 2.2. Inclusion and Exclusion Criteria

Inclusion criteria were as follows: meet the diagnostic criteria of pneumonia [8], with pathologic changes such as patchy infiltrating shadow and interstitial pneumonia by clinical imaging examination, 2–6 years old, and with well-documented clinical data.

Exclusion criteria were as follows: with bronchial dysplasia or congenital heart disease; with sepsis, malignancy, liver and kidney disease, or aspiration pneumonia; with familial diseases; and with blood system disease or congenital abnormal blood coagulation system.

### 2.3. Methods

#### 2.3.1. Sample Collection

Fasting venous blood (3 mL) was collected from all enrolled children in the morning and centrifuged at 2500 r/min at 4°C for 15 min. The upper yellow plasma was absorbed into EP tubes and stored in a refrigerator at 80°C.

#### 2.3.2. Detection of the Levels of Platelet miR-223 and miR-192

The total RNA in serum was extracted by TRIzol (Invitrogen, USA), and an ultraviolet spectrophotometer was used to detect the quality concentration and purity of RNA. Ensure no doping of phenol or protein. Reverse transcription was then performed with miR-223 (forward: 5′-TCCGAAGTGTACCTCAAC-3′, reverse: 5′-GTGCAGGGTCCGAGGT-3′) and miR-192 (forward: 5′-GGGGCTGACCTATGAATTGA-3′, reverse: 5′-CAGTGCAGGGTCCGAGGT-3′) reverse transcriptional primers. U6 (forward: 5′-CTCGCTTCGGCAGCACATATACT-3′, reverse: 5′-ACGCTTCACGAATTTGCGTGTC-3′) was used as internal reference. Then, fluorescence quantitative PCR instrument was used for amplification. The relative levels of miR-223 and miR-192 were calculated by the 2^△△CT^ method.

#### 2.3.3. Detection of Coagulation Function

The PT, APTT, and FIB in SP children were detected by the Sysmex CA-1500 System (Sysmex Corporation, Japan).

### 2.4. Statistical Methods

Data analysis was performed by SPSS, version 22. Qualitative data were expressed with (*n*, %) and analyzed by the *χ*^2^ test; quantitative data were expressed as mean ± SD ($\bar{x}\pm s$) and analyzed by the *t*-test. The Pearson analysis was conducted to evaluate the correlation between expression levels of miR-223 and miR-192 and coagulation function index in SP children. Differences were considered significant at *P* < 0.05.

## 3. Results

### 3.1. miR-223 and miR-192 in the Study Group and Control Group

miR-223 was significantly higher than that in the control group, and miR-192 was significantly lower than that in the control group (*P* < 0.05), as given in Table 1.

### 3.2. miR-223 and miR-192 in Different Infection Groups

Compared with the mild infection group, miR-223 was significantly higher and miR-192 was significantly lower in the moderate infection group and severe infection group (*P* < 0.05), as given in Table 2.

### 3.3. The Coagulation Function Indicators in the Study Group and Control Group

Compared with the control group, PT and APTT were significantly lower and FIB was significantly higher in the study group (*P* < 0.05), as given in Table 3.

### 3.4. The Coagulation Function Indicators in Different Infection Groups

Compared with the mild infection group, PT and APTT were significantly higher and FIB was significantly higher in the moderate infection group and severe infection group (*P* < 0.05), as given in Table 4.

### 3.5. Correlation between miR-223 and miR-192

Pearson correlation analysis revealed that miR-223 was negatively correlated with miR-192 (*r* = 0.253, *P* < 0.001), as shown in Figure 1.

### 3.6. Correlation Analysis of miR-223 and miR-192 with Coagulation Function

Pearson correlation analysis revealed that miR-223 was positively correlated with PT and APTT and negatively correlated with FIB (*P* < 0.05); miR-192 was negatively correlated with PT and APTT and positively correlated with FIB (*P* < 0.05), as given in Table 5.

## 4. Discussion

SP is a common condition in pediatric intensive care unit (ICU) which develops mainly from mild pneumonia. It is dangerous and develops rapidly, with the incidence rate increasing by about 13% every year [9]. Children SP is a critical disease with severe infection inside and outside the lungs and systemic organ involvement. Common symptoms include respiratory failure, systemic poisoning symptoms, other viscera function insufficient, and even sepsis [10]. Due to the incomplete development of the immune system in children, the pathogenic bacteria propagate rapidly and transmit through direct diffusion and blood flow, thus resulting in rapid deterioration into severe pneumonia [11]. Previous research has established that when the body is seriously infected, it will stimulate the release of inflammatory mediators and inflammatory cells in the body [12]. The released inflammatory factors can cause fibrinolysis or coagulation system disorders, the formation of thrombus in the microcirculation, and even disseminated intravascular coagulation (DIC), which seriously threatens the life and health of patients. Therefore, accurate diagnosis of SP in children and monitoring of coagulation function can provide a basis for early screening of children with poor prognosis. CRP, PCT, and blood cell analysis are indicators commonly used in the evaluation of SP, but have poor specificity, and the efficacy of prognostic assessment is also poor. Therefore, it is of great significance to search for more effective markers to evaluate the severity and prognosis of severe pneumonia.

In this study, miR-223 in the moderate infection group and severe infection group was significantly increased, and miR-192 was significantly decreased (*P* < 0.05) when compared with the mild infection group. It indicated that miR-223 and miR-192 were correlated with the severity of the disease. miRNA, a class of endogenous RNA molecules with length of 21–25 nt, participated in gene transcription regulation and is a key factor of signal transduction in and out of cells. miRNA regulates most of the genes and employed in various cellular processes such as cell proliferation, differentiation, metabolism, and apoptosis [13]. Currently, miRNA has been used as biomarker for disease diagnosis in many clinical fields, such as cardiovascular and cerebrovascular diseases, autoimmune diseases, and tumors [14, 15]. Studies have shown that miR-223 is highly expressed in peripheral blood of SP patients and can be used as an early diagnostic marker for severe pneumonia [16]. miRNA-192 is a primate-specific miRNA key to the occurrence, development, metastasis, and insulin resistance of tumors [17]. Previous research has established miRNA-192 as a biomarker for diagnosis of disease because that miRNA is unaffected by endogenous RNA enzymes and exists the peripheral blood system and tissue cells. Previous studies have confirmed that miR-223 can be used as a potential diagnostic marker of tuberculosis, and miR-192 can be used to assess the severity of disease in children with associated pneumonia [18]. It was demonstrated that miR-223 was significantly higher and miR-192 was significantly lower when compared with the control group (*P* < 0.05).

Among the coagulation indicators, APTT mainly detects endogenous coagulation and PT detects exogenous coagulation. FIB, an acute reaction protein, is the coagulation factor with the largest plasma content in the human body, and its level can indicate that blood is in high energy state [19]. Studies have shown that FIB is a risk factor for thrombosis and can be used as a predictor of the severity of pulmonary embolism [20]. It was demonstrated that PT and APTT in the study group were significantly lower than those in the control group, while FIB in the control group was higher than those in the control group (*P* < 0.05), indicating the hypercoagulable state. Compared with the mild infection group, APTT and PT in the moderate infection group and severe infection group were significantly increased, and FIB was significantly decreased (*P* < 0.05). It suggested that coagulation function was closely correlated with the severity of the disease. Pearson correlation analysis revealed that miR-223 was positively correlated with PR and APTT and negatively correlated with FIB (*P* < 0.05); miR-192 was negatively correlated with PR and APTT and positively correlated with FIB (*P* < 0.05). It suggested a close relationship between miR-223, miR-192, and coagulation.

## 5. Conclusion

Serum levels of miR-223 and miR-192 in platelet can reflect the severity the coagulation function in children with SP, which can provide a certain reference basis for clinical guidance and treatment and prognosis.

## Figures and Tables

**Figure 1:** Correlation between miR-223 and miR-192.

**Table 1:** miR-223 and miR-192 in the study group and control group ($\bar{x}\pm s$).

	miR-223	miR-192
Study group (*n* = 129)	2.28 ± 0.39	0.62 ± 0.18
Control group (*n* = 129)	1.67 ± 0.29	0.90 ± 0.24
*t*	14.490	10.600
*P*	<0.001	<0.001

**Table 2:** miR-223 and miR-192 in different infection groups ($\bar{x}\pm s$).

	miR-223	miR-192
Mild infection group (*n* = 43)	1.93 ± 0.31	0.93 ± 0.25
Moderate infection group (*n* = 43)	3.01 ± 0.49^a^	0.57 ± 0.23^a^
Severe infection group (*n* = 43)	3.67 ± 0.52^a^	0.47 ± 0.23^a^
*F*	164.100	44.870
*P*	<0.001	<0.001

Compared with the mild infection group, ^a^*P* < 0.05.

**Table 3:** The coagulation function indicators in the study group and control group ($\bar{x}\pm s$).

	PT (s)	APTT (s)	FIB (g/L)
Study group (*n* = 129)	10.90 ± 0.75	31.67 ± 1.25	3.94 ± 0.53
Control group (*n* = 129)	14.51 ± 1.04	35.64 ± 1.42	2.79 ± 0.31
*t*	31.980	23.830	21.270
*P*	<0.001	<0.001	<0.001

**Table 4:** The coagulation function indicators in different infection groups ($\bar{x}\pm s$).

	PT (s)	APTT (s)	FIB (g/L)
Mild infection group (*n* = 43)	14.13 ± 1.01	34.25 ± 1.28	3.16 ± 0.57
Moderate infection group (*n* = 43)	12.87 ± 0.89^b^	32.56 ± 1.25^b^	3.45 ± 0.56^b^
Severe infection group (*n* = 43)	10.21 ± 0.66^b^	31.45 ± 1.22^b^	3.77 ± 0.57^b^
*F*	229.800	54.690	12.470
*P*	<0.001	<0.001	<0.001

Compared with the mild infection group, ^b^*P* < 0.05.

**Table 5:** Correlation analysis of miR-223 and miR-192 with coagulation function.

	miR-223		miR-192	
	*r*	*P*	*r*	*P*
PT	0.592	<0.001	−0.645	0.237
PT	0.416	0.016	−0.711	0.188
FIB	−0.603	0.003	0.653	<0.001

## Data Availability

No data were used to support this study.
